# Increased miR-188-3p in Ovarian Granulosa Cells of Patients with Polycystic Ovary Syndrome

**DOI:** 10.1155/2021/5587412

**Published:** 2021-04-15

**Authors:** Beibei Dai, Jun Jiang

**Affiliations:** ^1^Department of Ultrasound, Obstetrics and Gynecology Hospital of Fudan University, 419 Fangxie Road, Shanghai 200011, China; ^2^State Key Laboratory of Genetic Engineering, School of Life Sciences, Fudan University, Shanghai 200438, China

## Abstract

MicroRNA-target networks are often dysregulated in diseases. Our purpose is to investigate this dysregulation of polycystic ovary syndrome (PCOS). Through the bioinformatics reanalysis of the public RNAseq dataset, we found that miR-188-3p was the miRNA with the highest induction rate, and indicated that miR-188-3p might have a rare function of upregulating its targeted expression. This discovery will increase our understanding of the pathology of PCOS and provide new targets for treatment strategies.

## 1. Introduction

Polycystic ovarian syndrome (PCOS) is a hormonal disease common in women of reproductive age [1]. The prevalence of PCOS, following the Rotterdam diagnostic criteria, in a meta-analysis of 15 studies is 10% [2]. Women with PCOS may have fewer or longer menstrual periods or have high-level male hormones (androgens), resulting in the ovaries accumulating many small amounts of fluid (follicles) and not releasing eggs regularly [3]. Signs and symptoms of PCOS usually develop around the first monthly period of puberty but can also appear after puberty as the gain of weight. The signs and symptoms of PCOS vary, such as irregular menstrual cycles, excessive androgens, and polycystic ovary. Complications of PCOS include infertility, gestational diabetes, miscarriage, premature birth, metabolic syndrome, abnormal uterine bleeding, and endometrial cancer and bring serious distress to the majority of women [4, 5]. PCOS is caused by many factors, including excessive insulin, low inflammation, heredity, and excessive androgens. However, it is not clear what is the most important pathogenic factor, which brings great difficulties to clinical treatment [6–8].

Although the pathological mechanism of PCOS has been clarified, the effect of miRNAs on the proliferation of ovarian granulosa cells remains to be further studied [4]. MiRNAs are short, noncoding RNAs that contain approximately 22 nucleotides [9, 10]. They can regulate messenger RNA (mRNA) expression by binding to complementary nucleotides on the 3′-UTR of the target mRNA. MiRNAs affect the physiological and pathological states of cells by regulating various cellular processes such as cell proliferation, cell differentiation and apoptosis, biosynthesis, and hormone secretion. Pioneers have studied how miRNAs regulate cells and influence the corresponding pathology. For example, recent evidence shows that miR-21, miR27b, miR-103, and miR-155, which are related to human obesity, have clear upregulation in women [11]. Besides, in mouse PCOS models, the enhancement of miR-21 and miR-146a is demonstrated to have a potential for DNA damage [12]. Previous studies have also performed miR-222 in membrane cells and found that miR-222 expression can be inhibited by androgens and targeted by cyclin-dependent kinase inhibitor 1B (p27Kip1), in order to regulate cell proliferation [13]. Subsequent studies on mir-222 have shown that it can reduce estrogen receptor alpha (ER*α*) protein levels, related signaling pathways, and targeted gene expression. However, miRNA implication in PCOS is still far from understood. In this bioinformatics study, we investigate miRNAs and their targets dysregulated in PCOS through the reanalysis of public RNAseq datasets. This study will bring more insights into the pathogenesis of PCOS and potentially provide new strategies for its therapy.

## 2. Materials and Methods

### 2.1. Data Resource

GEO DataSets were downloaded from https://www.ncbi.nlm.nih.gov/geo/ via accession numbers GSE138572 and GSE138518.

### 2.2. Differential Expression miRNA Analysis

Raw read counts were extracted from GEO DataSets. The miRNAs were preexcluded if their maximal read counts among all samples were no more than 5. Batch effect was corrected to make sure the samples with largely variable total read are comparable, using the correction method ComBat and the normalization method TMM. After the batch effect was corrected, PCOS samples were compared with control samples using DESeq2 [14]with the mean fit type and LRT test type via DEBrowser [15].

### 2.3. Differential Expression mRNA Analysis

Raw read counts were extracted from GEO DataSets. The mRNAs were preexcluded if their maximal read counts among all samples are no more than 100. PCOS samples were compared with control samples using DESeq2 [14] with the mean fit type and LRT test type via DEBrowser [15].

### 2.4. Collection of Predicted and Validated miRNA Targets

Targets of miRNA were bioinformatically predicted using miRDB (http://mirdb.org), TargetScan (http://www.targetscan.org/vert_72/), and DIANA (http://www.microrna.gr/microT-CDS). Experimentally validated miRNA-target interactions were collected from miRTarBase (http://miRTarBase.cuhk.edu.cn/).

### 2.5. Gene Set Enrichment Analysis (GSEA)

Predicted or validated miRNA targets by various algorithms were used to create gmx file. All mRNAs ranked by differential expression statistic were used to create rnk file. The miRNA targets were analyzed to test whether they were enriched in differentially expressed genes using GSEA software [16].

### 2.6. Overrepresentation Analysis

The selected gene list was analyzed for their overrepresentation in pathways of various databases and gene sets of many published datasets using Enrichr (http://amp.pharm.mssm.edu/Enrichr).

## 3. Results

### 3.1. miR-188-3p Was Upregulated in PCOS Tissues

To survey the miRNome dysregulation in PCOS, we extracted raw read count data from a publicly available dataset (GSE138572) which included ovarian granulosa cells isolated from five PCOS patients and five healthy controls. Two samples (one from the PCOS group and the other from the controls) had 14.4M and 6.1M total annotated reads, respectively, which were much higher than other samples (2.4M reads on This read count bias created a strong variance that cannot be adjusted by normalization. Therefore, we treated these two samples as the batch effect, which was corrected using the SVA's ComBat algorithm [17]. After correction, PCOS samples could be separated from controls based on miRNome using the principal component analysis (PCA; Figure 1(a)), with one minor exception. Next, we used DESeq2 via DEBrowser to analyze the fold change (FC) and the adjusted significance (*P*_adj_) of each miRNA between PCOS and controls. As shown in the volcano plot (Figure 1(b)), most miRNAs had a nonsignificant change in granulosa cells of PCOS (grey dots), except that miR-188-3p was significantly upregulated in PCOS (the red dot). This miRNA was barely expressed in granulosa cells of healthy women but induced in those of PCOS patients (Figure 1(c)).

### 3.2. Predicted Targets of miR-188-3p Were Upregulated in PCOS Tissues

Since miR-188-3p was a unique miRNA that showed significant dysregulation in ovarian granulosa cells of PCOS patients, we hypothesized that its mRNA targets might be downregulated in PCOS. We surveyed the predicted targets of miR-188-3p using three commonly used algorithms: miRDB [18], TargetScan [19], and DIANA [20]. Then, we used the target lists to create the gmx file for GSEA. In the meantime, we extracted raw read count data from a publicly available mRNAseq dataset (GSE138518) which included ovarian granulosa cells isolated from three PCOS patients and three healthy controls, and used DESeq2 via DEBrowser to analyze the statistic representing the confidence of fold change. The genes with their ranked statistic were used to create the rnk file for GSEA. Both the gmx file and the rnk file were input to GSEA software to evaluate how miR-188-3p target genes were distributed within the ranked differentially expressed genes. Surprisingly, miR-188-3p target genes predicted by either miRDB (Figure 2(a)) or DIANA (Figure 2(b)) were more frequent at top of the ranked list, indicating that they are generally upregulated. The target list predicted by TargetScan was excluded by the GSEA algorithm itself. These data suggest that miR-188-3p functions as an uncommon expression activator, rather than a canonical expression inhibitor, in ovarian granulosa cells.

### 3.3. Validated Targets of miR-188-3p Were Upregulated in PCOS Tissues

To further confirm our unexpected observation, we expanded GSEA analysis to experimentally validated miR-188-3p targets, which were surveyed from the miRTarBase [21]. The full gene list, as well as its subset (genes validated by HITS-CLIP or PAR-CLIP), was used to create the gmx files. Similar to the predicted targets, experimentally validated miR-188-3p targets were also enriched in the top of the ranked differentially expressed genes, based on the whole validated target list (Figure 3(a)), HITS-CLIP validated list (Figure 3(b)), or PAR-CLIP validated list (Figure 3(c)). Gene lists validated by other experimental approaches were excluded from the GSEA analysis due to their limited gene numbers. These data again support the finding that miR-188-3p upregulates the expression of targets.

### 3.4. Upregulated miR-188-3p Targets Were Enriched in PCOS Pathways

To explore the potential functions of genes upregulated by miR-188-3p in ovarian granulosa cells, we selected the targets that contributed to the core enrichment from the full experimentally validated targets via miRTarBase. Next, we performed the classical pathway analysis of this gene subset using Enrichr [22]. First, we confirmed that these genes are involved in PCOS pathology, as they were also overrepresented in the genes upregulated in PCOS endometrium (GSE48301) [23] from the disease perturbation database (Figure 4(a)). Second, these genes were responding to estradiol (Figure 4(b)) [24] [25], which was consistent with the fact that hormone imbalance is an important aspect of PCOS. Third, the upregulated miR-188-3p targets were enriched in adipogenesis (Figure 4(c)) using WikiPathways database [26], suggesting their implication in weight gain, a common symptom in PCOS patients. And last, these target genes were enriched in the canonical NF-*κ*B pathways (Figure 4(d)) using the NCI-Nature database [27], providing insights into the potential molecular mechanism of function.

## 4. Discussion

Several miRNAs have been reported to be dysregulated in PCOS ovaries [28]. miR-9 and miR-18b are found to be upregulated in PCOS and change the release of testosterone, progesterone, and estradiol via targeting IL8, SYT1, and IRS2 [29, 30]. Upregulation of miR-93 in adipose tissue of PCOS patients is found to alter hormone metabolism by targeting GLLU4 [31]. Dysregulation of miR-320 is found to affect estradiol production and release through the regulation of RAB5B, E2F1, and SF-1 expression [32, 33]. And the expression of miR-483-5p is affected in PCOS to change granulose cell proliferation by targeting Notch3, MAPK3, and IGF1 [34, 35]. However, these miRNAs show no significant difference in the cohort we analyze, likely due to the limited sample size.

Previously, miR-188-3p has been reported to be involved in various physiologic and pathological processes. Upregulation of miR-188-3p is reported to strongly associate with poor prognosis and short survival in two cohorts of colorectal cancer and may promote cancer cell migration by direct interaction with MLLT4 [36]. Downregulation of miRNA-188-3p is found to contribute to apoptosis of spermatogenic cells in patients with azoospermia by its regulatory role of MLH1 expression [37]. A study of cardiovascular diseases reveals that miR-188-3p suppresses autophagy and myocardial infarction by targeting ATG7 [38]. miR-188-3p is also found to have an inhibitory effect on macrophage inflammatory response and oxidation [39]. Nevertheless, the current study for the first time implicates miR-188-3p in PCOS.

The canonical function of miRNAs is to downregulate the expression of target mRNA, either via mRNA degradation or translational inhibition. However, some miRNAs have been found to upregulate targets in specific cells [10]. The translation activation function of miRNA was first discovered by Vasudevan et al. in the context of the cell cycle [40]. Later, liver-specific miR-122 was shown to activate hepatitis C virus (HCV) RNA expression through recruiting factors involved in RNA replication and translation, as well as increasing RNA stability [41–43]. The wildly expressed miR-10a was reported to interact with ribosomal protein mRNAs and enhance their translation, resulting in the elevation of global protein synthesis and thus cell transformation [44]. Our results in the current study suggest that miR-188-3p performs its regulatory function in such an uncommon way of upregulation in human ovarian granulosa cells, which warrants experimental validation in further studies.

In PCOS, miR-188-3p was found to regulate adipogenesis, which was frequently observed in patients. Approximately 50% of PCOS patients are overweight or obese [45]. Obesity increases insulin resistance and compensatory hyperinsulinemia, which in turn increases adipogenesis and decreases lipolysis. Obesity also induces insulin resistance and compensatory hyperinsulinemia, glucose intolerance, and dyslipidemia and increases the risk of pregnancy complications [46]. PCOS women with obesity have more severe phenotypes than the ones without obesity, including worse menstrual irregularity, infertility, miscarriage, prematurity, pregnancy-induced hypertension, gestational diabetes, biochemical and clinical hyperandrogenism, glucose intolerance and/or T2DM, and metabolic syndrome [47]. Regulated targets of miR-188-3p in PCOS were also enriched in the NF-*κ*B pathway, suggesting chronic inflammation involved [48, 49]. Consistently, the phosphatidylinositol 3-kinase/AKT/NF-*κ*B signaling pathway was reported to mediate WNT5a-induced inflammation and oxidative stress in ovarian granulosa cells in PCOS [50]. Furthermore, iridoids (a NF-*κ*B inhibitor) with genipin stem nucleus were proposed to protect PCOS patients from inflammatory damage [51]. All these pathway analyses could guide the further experimental investigation on the molecular mechanism of miR-188-3p implication in PCOS.

In summary, we reanalyzed miRNAseq and mRNAseq data from ovarian granulosa cells of PCOS patients or healthy controls and identified strong upregulation of miR-188-3p. In PCOS, miR-188-3p uncommonly induced, rather than inhibited, its predicted and validated mRNA targets, causing potential altered disease-related pathways.

Gene list for over-representation analysis:

- FPR1
- BTG2
- PTAFR
- SPIN3
- C3orf38
- SCN9A
- BACH1
- C3orf52
- METTL16
- MCU
- NUP98
- ZNF207
- SLC2A9
- CISD1
- NDUFA7
- TSC22D2
- CYLD
- ZNF350
- RAPGEF6
- NUFIP2
- NNT
- MCFD2
- KLF7
- HAS2

## Figures and Tables

**Figure 1:** miR-188-3p was upregulated in PCOS: (a) PCA analysis based on miRNome; (b) volcano plot screening for miRNAs with large fold change (FC) and strong significance (*P*_adj_); (c) corrected read counts of miR-188-3p between PCOS and controls.

**Figure 2:** Predicted targets of miR-188-3p were upregulated in PCOS: (a) miR-188-3p targets predicted by miRDB; (b) miR-188-3p targets predicted by DIANA.

**Figure 3:** Validated targets of miR-188-3p were upregulated in PCOS: (a) all experimentally validated miR-188-3p targets collected in miRTarBase; (b) miR-188-3p targets validated by HITS-CLIP; (c) miR-188-3p targets validated by PAR-CLIP.

**Figure 4:** Pathway analysis of the validated miR-188-3p targets contributing to core enrichment of GSEA. Overrepresentation analysis was performed using the Enrichr against disease perturbation database (a), ligand perturbation database (b), human WikiPathways database (c), and NCI-Nature database (d). Color code represents the *P* value.

## Data Availability

The datasets used and/or analyzed during the current study are available from the corresponding author on reasonable request.
